The article "Influences of Magnetic Resonance Imaging Superresolution Algorithm-Based Transition Care on Prognosis of Children with Severe Viral Encephalitis" was published in 2022. Journal: Comput Math Methods Med.

# Influences of Magnetic Resonance Imaging Superresolution Algorithm-Based Transition Care on Prognosis of Children with Severe Viral Encephalitis

**DOI:** 10.1155/2022/5909922

**Published:** 2022-06-17

**Authors:** Yan Wang, Yan Zhang, Ling Su

**Affiliations:** Department of Infusion Room of Emergency, Children's Hospital of Nanjing Medical University, Nanjing, 210000 Jiangsu Province, China

## Abstract

**Objective:**

Its goal was to see how convolutional neural network- (CNN-) based superresolution (SR) technology magnetic resonance imaging- (MRI-) assisted transition care (TC) affected the prognosis of children with severe viral encephalitis (SVE) and how effective it was.

**Methods:**

90 SVE children were selected as the research objects and divided into control group (39 cases receiving conventional nursing intervention) and observation group (51 cases performed with conventional nursing intervention and TC intervention) according to their nursing purpose. Based on SR-CNN-optimized MRI images, diagnosis was implemented. Life treatment and sequelae in two groups were compared.

**Results:**

After the processing by CNN algorithm-based SR, peak signal to noise ratio (PSNR) (40.08 dB) and structural similarity (SSIM) (0.98) of MRI images were both higher than those of fully connected neural network (FNN) (38.01 dB, 0.93) and recurrent neural network (RNN) (37.21 dB, 0.93) algorithms. Diagnostic sensitivity (95.34%), specificity (75%), and accuracy (94.44%) of MRI images were obviously superior to those of conventional MRI (81.40%, 50%, and 80%). PedsQLTM 4.0 scores of the observation group 1 to 3 months after discharge were all higher than those of the control group (54.55 ± 5.76 vs. 52.32 ± 5.12 and 66.32 ± 8.89 vs. 55.02 ± 5.87). Sequela incidence in the observation group (13.73%) was apparently lower than that in the control group (43.59%) (*P* < 0.05).

**Conclusion:**

(1) SR-CNN algorithm could increase the definition and diagnostic ability of MRI images. (2) TC could reduce sequelae incidence among SVE children and improve their quality of life (QOL).

## 1. Introduction

Viral encephalitis is an inflammatory lesion of the brain parenchyma mainly caused by viral infection, including herpes simplex virus, arbovirus, and other common viruses. It is the commonest disease among children [1, 2]. Viral encephalitis is featured with sudden onset, rapid development, and high mortality, especially severe viral encephalitis (SVE) [3]. Children with SVE usually suffer from epilepsy, mental retardation, paralysis, dyskinesia, and other sequelae, which cause huge burden to families. Therefore, definite diagnosis and out-of-hospital care are very important for SVE children [4].

According to several research, a thorough systematic nursing intervention (mental nursing and rehabilitation guidance) for children with SVE sequela after discharge could enhance their prognosis and quality of life (QOL) [5]. Based on the preceding findings, American specialists propose transition care (TC). TC was aimed at enabling patents to receive collaborative and transition care on different sites [6]. TC focuses on long-term nursing and enhances the self-care abilities of patients and their family members under the guidance of evidence-based basis. Besides, it was shown that TC mode can evidently enhance functional activities, compliance, and QOL of patients [7]. TC mode is gradually developed towards China. At present, the study on the application of TC focuses mainly on postpartum [8] and chronic diseases [9]. The studies on its application in SVE sequela among children.

In terms of the diagnosis of viral encephalitis, imaging technologies currently show good application values. Magnetic resonance imaging (MRI) is one of them [10]. It is proposed in a large number of studies that MRI examination demonstrates significant clinical application values in the diagnosis and differential diagnosis of viral encephalitis in children [11, 12]. In addition, MRI images possess high resolution. However, an MRI image with higher resolution indicates longer acquisition time and higher requirement for devices due to hardware, physical, and physiological limitations. With the studies in recent years, superresolution (SR) technology is put forward. SR technology assesses low resolution (LR) images and then transmits the result to high resolution (HR) images to minimize the error between HR images and original images [13]. With the emergence of deep learning (DL), SR technology is further optimized [14]. Convolutional neural network (CNN) algorithm is a widely applied SR technology. Relevant studies reveal that CNN algorithm shows excellent performance in image processing [15].

CNN-based SR technology (SR-CNN) was adopted to optimize MRI images, assist TC in carrying out the prognosis and nursing of SVE children, and assess the application effects on the improvement of SVE sequela among children, which are aimed to provide more effective therapeutic and nursing methods for the children with viral encephalitis, reduce the incidence of SVE sequela, and improve the daily QOL of SVE children.

The following is the paper's organization paragraph: In Section 2, the research method is provided. The experimental results are examined in Section 3.  Section 4 consists of the discussion section. Finally, the research job is completed in Section 5.

## 2. Research Methods

### 2.1. Research Objects

A total of 90 SVE youngsters were chosen as research subjects, with 49 boys and 41 females hospitalised to our hospital between March 2020 and March 2021. Their average age was between 5 and 14 with the average of 8.98 ± 1.08. There were 78 children with clinical fever, 26 with vomiting, 58 with convulsion, 31 with coma, 12 with limb disorder, 23 infected by herpes simplex virus, 31 with infected by adenovirus, 19 infected by cytomegalovirus, and 11 for other reasons. The children were divided into two groups depending on the intentions of the children and their families: control group (39 cases with typical nursing intervention after discharge) and observation group (51 cases receiving TC intervention based on conventional nursing). SR-CNN-based MRI images were utilized to diagnose the patients in two groups. Besides, the prognosis of the two groups was compared. The implementation of the research had been approved by relevant Medical Ethics Committee.

The patients were included based on the following standards.

- All children could engage in the research and communication with certain understanding ability
- Children's parents did not suffer from cognitive or speech dysfunction
- Children volunteered to participate in the research and had signed informed consent
- All children conformed to the standard of viral encephalitis in *neurology* [16]

The patients were excluded based on the following standards.

- Children themselves sufferer from other central nervous diseases or chronic diseases
- Children suffered from severe epidemic encephalitis type B
- Children did not participate in a complete study

### 2.2. CNN Algorithm-Based SR Technology

CNN algorithm currently shows good application effects in various fields. As a feedforward neural network (FNN), CNN mainly consists of three components, including convolutional layer, pooling layer, and fully connected layer, as shown in Figure 1.

Convolutional layer is made up of convolution kernel and activation function. Its main function is the extraction of the features of target images. Convolutional kernel recognizes the features of images, and activation function obtains multidimensional images. The specific calculation method is shown as follows:

(1) $$\begin{array}{c} S=\int_{L}^{L-1}\int_{W}^{W-1}P•\omega +b. \end{array}$$

In equation (1), *P* represents the input target image. *S* refers to the output image. *L* and *W* denote the length and width of the image, respectively. *ω* stands for convolutional kernel. *b* represents bias. *•* is the convolution operation. In convolutional layer, the convolution operation is performed on *P* and *ω* according to bitwise multiplication. The calculation method is expressed as follows:

(2) $$\begin{array}{c} S^{\prime }=Q_{1}\times \omega +Q_{2}\times \omega +\cdots +Q_{n}\times \omega . \end{array}$$

In equation (2), *Q* represents the image region, *n* refers to the number of regions, and *S*′ denotes the output convolution feature diagram.

The main function of the pooling layer is the sampling of feature images to reduce training parameters as well as computation and avoid overfitting. The pooling layer is mainly divided into maximum pooling layer and average pooling layer.  Figure 2 demonstrates the specific calculation process.

The white region in Figure 2 is set as the example. The pooling process of the average is expressed as follows:

(3) $$\begin{array}{c} P^{\prime }=\frac{p4+p5+p5+p6}{4}. \end{array}$$

The above equation is simplified as follows:

(4) $$\begin{array}{c} \frac{4+5+5+6}{4}=5. \end{array}$$

The pooling process of the maximum is expressed as follows:

(5) $$\begin{array}{c} P^{\prime }=\left\{p4<p5=p5<p6\right\}P^{\prime }=p_{\max}. \end{array}$$

The above equation is simplified as follows:

(6) $$\begin{array}{c} P^{\prime }=6\left(4<5=5<6\right). \end{array}$$

In equation (6), *P*′ represents the pooling value of output image features, *p* denotes the pooling value in the picture of an image region, and *P*_max_ refers to the maximum.

The main function of fully connected layer is the connection of all feature images and the classification of these images to obtain the results by classifier.

In image reconstruction, SR technology reversely obtains HR images from LR images. The key step is upsampling, which is also the main action step of CNN algorithm. The upper sampling layer is divided into preupsampling (the images of the same size as target images are obtained from LR images, and their features are extracted, and their display effects are enhanced), postupsampling (the size of input images is kept the same), progressive upsampling (the reconstructed images are gradually enlarged to 2 times to obtain the images with different resolutions), and iterative up-down sampling (the features of HR images at different stages are obtained). According to the operation methods of upper sampling layer, it can also be divided into deconvolution layer and subpixel layer.

The main operation of deconvolution layer is enlargement-zero-padding-convolution. It is assumed that the original image *T* is *m* × *n*, enlarged image *T*′ is specifically expressed as follows:

(7) $$\begin{array}{c} T^{\prime }=\left(m+m\times 1\right)\times \left(n+n\times 1\right). \end{array}$$

The image *T*^″^ obtained by zero-padding is expressed as follows:

(8) $$\begin{array}{c} T^{\prime \prime }=\left(m+m\times 1+1\right)\times \left(n+n\times 1+1\right). \end{array}$$

Convolution refers to the convolutional image obtained by calculation according to CNN algorithm.

The main function of subpixel layer is the rearrangement of the image features obtained by convolution to acquire high-resolution images.

CNN algorithm-based SR image is assessed by peak signal to noise ratio (PSNR), structural similarity (SSIM), and its diagnostic efficacy.

(9) $$\begin{array}{c} \text{PSNR}=10*\log_{10}\left(\frac{{\left(2^{B}-1\right)}^{2}}{\left(1/mn\right)\sum_{i=0}^{m-1}\sum_{l=0}^{n-1}\left(C-U\right)}\right), \end{array}$$

where 2^*B*^ − 1 denotes the maximum pixel value of the image, *n* refers to the binary number of pixel value, *m* represents the number of image samples, *i* and *l* stand for certain pixel point in the image, *C* refers to clear image, and *U* means noisy image.

(10) $$\begin{array}{c} \text{SSIM}\left(C,U\right)=\frac{2\alpha_{C}\alpha_{U}+B}{{\alpha_{C}}^{2}+{\alpha_{U}}^{2}+B}, \end{array}$$

(11) $$\begin{array}{c} \alpha_{C}=\frac{1}{H\times W}\overset{H}{\underset{i=1}{\sum }}\overset{W}{\underset{l=1}{\sum }}C, \end{array}$$

(12) $$\begin{array}{c} \alpha_{U}=\frac{1}{H\times W}\overset{H}{\underset{i=1}{\sum }}\overset{W}{\underset{l=1}{\sum }}U, \end{array}$$

where *H* × *W* denotes the images size, *α* represents the average value, and *B* refers to the constant.

Greater PSNR and SSIM values indicate better processing effect on images.

### 2.3. MRI Examination

The examination of all children was performed by one magnetic resonance scanner and review by one surgeon. The films were reviewed by two experienced (20 years or more) clinicians. Siemens superconducting magnetic resonance scanner (model number was Magnetom Impct 1.0 T, spin echo, Germany) was adopted. The scanning parameters were set as follows. The thickness was 2.5 mm, layer-to-layer spacing was 3 mm, and time of repetition (TR) was 0.6 s and 3.4 s. Time of echo (TE) was 15 sm and 89 sm. Scanning planes included cross plane, sagittal plane, and coronal plane. Scanning sequences included T1WI and T2WI. The process of enhanced scanning was as follows. The contrast agent (Gd-DTPA, 0.2 mL/kg) was injected intravenously. The obtained images were processed by MRI and then optimized by CNN algorithm-based SR technology.

### 2.4. Nursing Methods

The children in the control group were performed with conventional nursing. The information about the patients' disease was obtained by phone 3 days after discharge, including diet, physical condition, and activity level. According to the obtained information, the corresponding nursing guidance was offered. The patients were told to visit outpatient department for review after 1 month and 3 months.

The children in the observation group received TC based on the nursing method for the control group. Firstly, a special TC team was composed of chief physicians, supervisor nurses, nursing graduates, therapists, and psychologists at pediatric department. Secondly, scales of pediatric quality of life inventory version 4.0 (PedsQL™ 4.0) [17] assessment was conducted on the patients before discharge and then set up health files, formulated discharge plans, and handed out record books to the patients' parents to prompt them to record their children's daily health status. Finally, to promote contact between patients' parents and medical nursing workers, a network video technique was used to provide SVE advice and training 2 to 3 weeks following discharge. Finally, the patients were informed that a follow-up visit would be scheduled one month after discharge. Besides, a target nursing scheme was formulated according to the result of the follow-up visit. Fifthly, home nursing guidance was carried out 2 months after discharge. Besides, psychological nursing intervention was performed according to the specific situations. Finally, the patients were informed of review 3 months after discharge, and nerve physique examination was also needed.

PedsQL™ 4.0 scores of the children in two groups at discharge, 1 month after discharge, and 3 months after discharge were compared. In addition, the incidence probability of patients' sequela (aphasia, acroparalysis, consciousness disorder, psychiatric disorders, dementia, epilepsy, deafness, impaired vision, and facial nerve numbness) 3 months after discharge was also compared.

### 2.5. Statistical Methods

The original data were input into the SPSS 22.0 statistical software for data analysis. Measurement data were expressed by mean ± standard deviation ($\bar{x}\pm s$). Independent sample *t*-test was used for pairwise comparison. Enumeration data were denoted by frequency and percentage (%). *χ*^2^ test was utilized for pairwise comparison. *P* < 0.05 indicated that the differences were statistically significant.

## 3. Results

### 3.1. Comparison of Algorithm Performance

MRI images of 3 children with viral encephalitis were used as the sample, and the optimization performance of CNN algorithm, fully connected neural network (FNN) [18], and recurrent neural network (RNN) [19] for SR technology was compared. The result showed that the average PSNR and SSIM values of MRI images processed by CNN algorithm-based SR technology were 40.08 dB and 0.98, respectively. Those processed by FNN algorithm-based SR technology were 38.01 dB and 0.93, respectively. Those processed by RNN algorithm-based SR technology were 37.21 dB and 0.93, respectively. According to the comparison, PSNR and SSIM of the images processed by CNN algorithm-based SR were both higher than those processed by FNN algorithm- and RNN algorithm-based SR, as Figure 3 illustrates.  Figure 4 displays the processing effects of three algorithms on images. It was demonstrated that MRI images processed by CNN algorithm-based SR technology showed higher definition.

### 3.2. Diagnostic Efficacy of SR Algorithm-Based MRI Images

According to the results of cerebral effusion examination, the diagnostic effect of MRI images on 90 included children with viral encephalitis was assessed and compared with that of conventional MRI images (the children diagnosed with viral encephalitis were positive, otherwise negative), as Tables 1 and 2. According to the calculation results, the diagnostic sensitivity, specificity, and accuracy of SR-CNN algorithm-based MRI images reached 95.34%, 75%, and 94.44%, respectively. Those of conventional MRI images amounted to 81.40%, 50%, and 80%, respectively. Apparently, the diagnostic efficacy of SR-CNN algorithm-based MRI images was superior to that of conventional MRI, indicating certain accuracy of the research.

### 3.3. Comparison of General Data

Figure 4 shows the statistical comparison of general clinical data on the patients in two groups. In terms of gender distribution, the proportions of male and female children in the control group were 53.85% and 46.15%, respectively. In the observation group, the proportions of male and female children reached 54.90% and 45.10%, respectively. The gender distribution in the two groups showed no remarkable statistical significance (*P* < 0.05). As for average age, the average age of the children in the control group was 8.12 ± 1.68, and that in the observation group amounted to 8.89 ± 0.99. The comparison of the average age between two groups revealed no notable statistical difference (*P* < 0.05). With respect to the distribution of clinical manifestations, the proportions of clinical manifestations of fever, vomiting, convulsion, coma, and limb disorders in the control group were 84.62%, 28.21%, 64.10%, 33.33%, and 12.82%, respectively. Those in the observation group were 88.24%, 23.53%, 64.71%, 35.29%, and 13.73%, respectively. The comparison indicated no evident statistical difference (*P* < 0.05). As to virus type distribution, the proportions of herpes simplex virus, adenovirus, cytomegalovirus, and other viruses in the control group reached 25.64%, 33.33%, 20.51%, and 10.26%, respectively. Those in the observation group amounted to 25.49%, 35.29%, 21.57%, and 13.73%, respectively. The comparison showed no statistical difference (*P* < 0.05). The above results suggested that the research was feasible to some extent.

### 3.4. PedsQLTM 4.0 Scores

Figure 5 displays the comparison of PedsQLTM 4.0 scoring results of the children in two groups at discharge, 1 month after discharge, and 3 months after discharge. There was no discernible difference in PedsQLTM 4.0 scores between control group (48.99 ± 4.91) and observation group (49.03 ± 4.32) at discharge (*P* < 0.05). PedsQLTM 4.0 scores of the children in the control group 1 month and 3 months after discharge were 52.32 ± 5.12 and 55.02 ± 5.87, respectively. Those in the observation group reached 54.55 ± 5.76 and 66.32 ± 8.89, respectively. PedsQLTM 4.0 scores in the two groups were both improved compared with those before discharge. Besides, PedsQLTM 4.0 scores of the observation group 1 month and 3 months after discharge were both superior to those of the control group (*P* < 0.05).

### 3.5. Incidence of Sequelae

Table 3 displays the incidence of various sequelae among the children in two groups. According to the calculations, the incidence of squeal in the control group was 43.59% percent, while it was 13.73% in the observation group. The incidence of squeal in latter group was apparently lower than that in former one (*P* < 0.05), as Figure 6 presents.

## 4. Discussion

With the development of current medical industry, the need for high-resolution images by the diagnosis and treatment of clinical diseases is becoming more and more urgent. Deep leaning method is of great significance to the reconstruction of SR images. Multiple research have suggested that deep learning-based neural network algorithms, particularly the CNN method, have considerable optimization impacts in the medical imaging SR field [20–22]. The processing effect of SR technology based on the CNN algorithm was compared to that of SR technology based on the FNN and RNN algorithms. The results demonstrated that PSNR (40.08 dB) and SSIM (0.98) of MRI images processed by CNN algorithm-based SR were both higher than those processed by FNN algorithm- (38.01 dB and 0.93) and CNN algorithm-based SR (37.21 dB and 0.93). MRI images processed by CNN algorithm-based SR showed the highest definition, which indicated that CNN algorithm improved the image reconstruction effects of SR technology very well. The result was consistent with the conclusions of most relevant studies [23, 24]. In addition, it was concluded that the diagnostic sensitivity (95.34%), specificity (75%), and accuracy (94.44%) of SR-CNN algorithm-based MRI images were obviously superior to those of conventional MRI (81.40%, 50%, and 80%). The conclusion revealed that SR-CNN algorithm-based MRI images could improve the diagnostic effect of MRI images, which was consistent with the outcomes of the studies conducted by Yan et al. [25] and Park et al. [26] and provided the basis for the accuracy of subsequent studies.

Based on the above research results, the effect of TC on children with SVE was investigated and compared with conventional nursing effect. It was pointed out in some studies that TC technology was not only very practical but also could reduce health care costs [27]. The systematic analysis of the consumption of health care costs was not involved in the research. However, the nursing effects of TC on QOL of SVE children after discharge and sequelae were compared. The results suggested that PedsQLTM 4.0 scores of the children in the observation group 1 month and 3 months after discharge were both superior to those in the control group (54.55 ± 5.76 vs. 52.32 ± 5.12 and 66.32 ± 8.89 vs. 55.02 ± 5.87). The incidence of sequelae in the observation group (13.73%) was obviously lower than that in control group (43.59%) (*P* < 0.05), which implied that reasonable and normative physiological and psychological nursing based on detailed record and understanding of children's disease was more conducive to the recovery of the children and reduced the incidence probability of sequelae among them. According to the study conducted by Chen et al. [28], TC exerted a profound influence on the nursing of stroke patients. Besides, it was put forward in multiple studies that TC was needed in the late care for many diseases [29]. Van et al. [30] also pointed out in their study that TC could not only effectively reduce medical system cost but also enhanced the effective rate of the treatment for patients and reduce patient readmission rate. The results of the above studies were all consistent with the research outcome and gave good support to the research.

## 5. Conclusion

After the examination on SVE patients with SR-CNN algorithm-based MRI images, TC was adopted to carry out prognostic care for SVE children. The results were as follows.

- SR-CNN algorithm could enhance the definition and diagnostic efficacy of MRI images
- TC could reduce the incidence of sequelae among SVE children and improved their QOL

Nonetheless, the impact of diagnostic accuracy on nursing effects was left out of the study, making it incomplete. As a result, more research was required. It could not be underestimated that the application of TC in sequela nursing for SVE children after discharge was advanced, and the application prospect was worth expectation.

## Figures and Tables

**Figure 1:** CNN action process (inside the yellow boxes are the captured feature images).

**Figure 2:** Pooling layer action process: (a) average pooling; (b) maximum pooling.

**Figure 3:** PSNR and SSIM results as well as the comparison of processing effects (the images in line 1 were taken from diagonal plane, those in line 2 were taken from transverse slope, and those in line 3 were taken from sagittal view).

**Figure 4:** Comparison of general data (A represents fever, B denotes vomiting, C refers to convulsion, D means coma, and E indicates limb disorders) (A represents herpes simplex virus, B denotes adenovirus, C refers to cytomegalovirus, and D stands for other viruses).

**Figure 5:** Comparison of PedsQLTM 4.0 scores (A represents PedsQLTM 4.0 scores at discharge, B denotes those 1 month after discharge, and C refers to those 3 months after discharge).

**Figure 6:** Comparison of incidence of sequelae.

**Table 1:** Diagnostic results of SR-CNN-based MRI images.

		Cerebral effusion examination (*n* = 90 cases)		Total
		Positive	Negative	
SR-CNN-based MRI (*n* = 90 cases)	Positive	82	01	83
	Negative	04	03	07
Total		86	04	90

**Table 2:** Diagnostic results of conventional MRI images.

		Cerebral effusion examination (*n* = 90 cases)		Total
		Positive	Negative	
Conventional MRI (*n* = 90 cases)	Positive	70	02	72
	Negative	16	02	18
Total		86	04	90

**Table 3:** Incidence of sequelae.

	Control group (*n* = 39 cases)	Observation group (*n* = 51 cases)	Total
Aphasia	04	01	05
Acroparalysis	02	01	03
Consciousness disorder	00	0	0
Psychiatric disorders	0	0	0
Dementia	01	0	01
Epilepsy	01	0	01
Deafness	02	02	04
Impaired vision	03	01	04
Facial nerve numbness	04	02	06
Total	17	07	24

## Data Availability

The datasets used and analyzed during the current study are available from the corresponding author on reasonable request.
